# Poly[(3-hexylthiophene)-*block*-(3-semifluoroalkylthiophene)] for Polymer Solar Cells

**DOI:** 10.3390/ijms11125027

**Published:** 2010-12-06

**Authors:** Ichiko Yamada, Koji Takagi, Yasuhiko Hayashi, Tetsuo Soga, Norio Shibata, Takeshi Toru

**Affiliations:** 1 Department of Frontier Materials, Graduate School of Engineering, Nagoya Institute of Technology, Gokiso, Showa-ku, Nagoya 466-8555, Japan; E-Mails: jade1cat@yahoo.co.jp (I.Y.); soga@nitech.ac.jp (T.S.); nozshiba@nitech.ac.jp (N.S.); 2 Department of Materials Science and Engineering, Graduate School of Engineering, Nagoya Institute of Technology, Gokiso, Showa-ku, Nagoya 466-8555, Japan; E-Mail: takagi.koji@nitech.ac.jp; 3 Department of Research, Nagoya Industrial Science Research Institute, 1-13 Yotsuyadori, Chikusa-ku, Nagoya 464-0819, Japan; E-Mail: tmtoru@mb.ccnw.ne.jp

**Keywords:** conjugated block copolymer, fluorine, semifluoroalkyl chain, PCBM, solar cell

## Abstract

We report the synthesis of poly[(3-hexylthiophene)-*block*-(3-(4,4,5,5,6,6,7,7,7-nonafluoroheptyl)thiophene)], P(3HT-*b*-3SFT), carried out by the Grignard Metathesis Method (GRIM). The copolymers composition was determined by ^1^H and ^19^F NMR spectroscopies, and gel permeation chromatography (GPC). The thin films of P(3HT-*b*-3SFT) were investigated by ultraviolet-visible absorption spectroscopy and atomic force microscopy (AFM). We also fabricated bulk-hetero junction (BHJ) solar cells based on blends of P(3HT-*b*-3SFT) and [6,6]-phenyl-C_61_-butyric acid methyl ester (PCBM). Although the composition ratio of P3SFT in P(3HT-*b*-3SFT) was low, the influence of P3SFT on the morphology and properties of solar cells was significant. The annealing process for the BHJ solar cells induced the formation of large domains and led to poor solar cell performance. The BHJ solar cells, based on PCBM and P(3HT-*b*-3SFT), prepared by the non-annealing process, had a maximum power conversion efficiency of 0.84% under 100 mW/cm^2^ (AM 1.5 solar illumination) in air.

## 1. Introduction

The bulk heterojunction (BHJ) solar cells, consisting of π-conjugated polymers as donor and fullerene derivatives as acceptor, have the advantage of low cost fabrication and easy processing due to solution based low temperature processes. The polymer-based solar cells have been attracting much attention and have been investigated by many researchers [1–7].

The mechanism by which organic thin-film solar cells convert sun-light into electricity is as follows. Absorption of photon leads to the formation of the electron-hole pair (exciton). Exciton diffuses to the interface of the donor and acceptor domains, where exciton is dissociated, that is, the charge separation occurs. The separated charges (free holes and electrons) are transported to the charge extracting electrodes through their respective transport materials (polymer and fullerene), to supply an external direct current [8].

The nanoscale morphology using the organic film as an active layer is an important factor in influencing the performance of the BHJ solar cells. The smaller phase domain of donor and acceptor materials has a larger interfacial area in the active layer, which leads to an efficient exciton separation. In addition, an interpenetrating and bicontinuous network of donor and acceptor materials allow the pathway to improve charge carrier conduction through the active layer to the respective electrodes. Various studies have been attempted to control the nanoscale-interpenetrating network of donor and acceptor materials in order to improve device performance. The character of spin-casting solvents and the additive in the solvents, affects phase segregation of two components [6,9,10]. The thermal annealing also controls the nanoscale organization and induces segregation of polymer and fullerene derivative [7,9]. The devices using donor-acceptor hybrid diblock copolymer have been studied [11–13]. In this study, we attempted to construct an interpenetrating networks structure of the donor and acceptor phase in the photoactive layer using, not only self-assembly of diblock copolymer, but also fluorine property.

It is well known that several diblock copolymers containing various conjugated segments self-assemble and form a nano-scale separated structure. This behavior improves the crystallinity of polymer film for organic electronic devices, so some diblock copolymers based on alkyl-thiophene were synthesized [14–17], and the organic devices have been fabricated [18,19].

On the other hand, the fluorine atom has the unique property of extremely low polarizability, which adds a lipophobic and hydrophobic nature to the fluorinated compounds, called “fluorophilic”. Due to the repelling nature of the fluorine to the non-fluorine compounds, the fluorine and non-fluorine phases are separated in the liquid state. This phenomenon is also observed in the hybrids of fluorinated and non-fluorinated elements in the solid state [20,21]. We report on diblock copolymers that consist of thiophenes with hydrocarbon and fluorinated carbon chains to construct the interpenetrating network structures of the donor and acceptor phase in the photoactive layer. We envisaged that in the active layer of solar cells composed of the diblock copolymer and fullerene derivative, the semifluoroalkyl segments would come close to each other by the intimate interaction among the alkylthiophene parts, and the repulsive effect between the semifluoroalkyl and alkyl groups. The fullerene derivatives would reside near the P3HT segments. A schematic image is shown in Figure 1.

The diblock copolymer, poly[(3-hexylthiophene)-*block*-(3-(4,4,5,5,6,6,7,7,7-nonafluoroheptyl) thiophene)] (P(3HT-*b*-3SFT)) we synthesized, consists of poly(3-hexylthiophene) (P3HT) and semifluoroalkyl chain-substituted polythiophene, poly(3-(4,4,5,5,6,6,7,7,7-nonafluoroheptyl)thiophene) (P3SFT). P3SFT has a spacer between the thiophene ring and the fluoroalkyl chain, which was expected to relieve the electron-withdrawing effect of the fluorine atoms and, hence, lower the oxidation potential of the thiophene ring, so that P3SFT has electronic properties similar to 3-alkylthiophenes [22]. The composition and characteristics of the diblock copolymer and the performance of the solar cells fabricated with P(3HT-*b*-3SFT):PCBM blend were studied.

## 2. Results and Discussion

### 2.1. Synthesis of Poly[(3-hexylthiophene)-*block*-(3-(4,4,5,5,6,6,7,7,7-nonafluoroheptyl)thiophene)], P(3HT-b-3SFT)

Diblock copolymer of P(3HT-*b*-3SFT) was synthesized from two monomers, 2,5-dibromo-3-(4,4,5,5,6,6,7,7,7-nonafluoroheptyl)thiophene (D3SFT) (5) and 2,5-dibromo-3-hexylthiophene (D3HT) (6), by the Grignard metathesis method (GRIM) [14,23,24]. D3SFT (5) were prepared by the methods reported previously [25] (Scheme 1). D3HT (6) was also prepared by bromination of 3-hexylthiophene [22]. The synthetic route for the P(3HT-*b*-3SFT) (10) is shown in Scheme 2. In the first step, the P3HT homopolymer (8) was synthesized, because the P3SFT homopolymer was immediately deposited from the polymerization system. In the second step, the GRIM product of D3SFT (9) was added to the reaction solution to give the diblock copolymer, P(3HT-*b*-3SFT) (10), where the feed molar ratio of D3SFT to D3HT was 50:100. P(3HT-*b*-3SFT), prepared in an increased ratio of the D3SFT, was deposited during the polymerization reaction, and the resulting copolymer was not dissolved in any of the solvents (e.g., THF, CHCl_3_ and ODCB).

We succeeded in the synthesis of two P(3HT-*b*-3SFT)s having different molecular weights by using a catalyst of 1.0 and 2.0 mol% Ni(dppp)Cl_2_. The P3HT homopolymer was also prepared as a reference by the same method described above.

### 2.2. Polymer Characterization

P3HT and P(3HT-*b*-3SFT)s were investigated by ^1^H NMR and ^19^F NMR spectroscopies. In the ^19^F NMR spectrum of P(3HT-*b*-3SFT), the fluorine signals indicate the semifluoroalkyl chain in diblock copolymer (Supplementary Figure S1; for convenience, only the diblock copolymer prepared by 2 mol% catalyst is shown). The compositions of both copolymers P(3HT-*b*-3SFT)s were determined from the integral ratio of the signals of P3HT and P3SFT in the ^1^H NMR spectrum. Supplementary Figures S2 and S3 show the ^1^H NMR spectra of P3HT and P(3HT-*b*-3SFT). The signal at 1.9–2.3 ppm appears only in the ^1^H NMR spectrum of P(3HT-*b*-3SFT). According to the ^1^H NMR spectrum of 3-(4,4,5,5,6,6,7,7,7-nonafluoroheptyl)thiophene [22], the signals are estimated corresponding to the β,γ-methylene protons of P3SFT. Thus, the ratios of the P3HT and P3SFT segments in P(3HT-*b*-3SFT)s, synthesized by using 1 mol% and 2 mol% Ni(dppp)Cl_2_ catalysts, were determined to be 100:3 and 100:12, respectively, on the basis of the signals corresponding to P3ST and P3SFT. The contents of P3SFT, however, do not correspond to the feed molar ratio of D3HTT:D3SFT = 100:50, showing that D3SFT is rather inactive toward the polymerization reaction and was not very involved in the polymer chain. In fact, the yield of P(3HT-*b*-3SFT)s was low (approximately 30% yield). It should be noted that the solubility of P(3HT-*b*-3SFT) in THF and CHCl_3_ was observed to be lower than P3HT itself, in spite of the low content of the 3-semifluorohepthlthiophene segment in P(3HT-*b*-3SFT)s.

The number-average (Mn) and the weight-average (Mw) molecular weight of diblock copolymers were measured by gel permeation chromatography (GPC) with THF as an eluent. Figure 2 shows the GPC profiles of P(3HT-*b*-3SFT)s, and the obtained molecular weights are integrated in Table 1. P(3HT-*b*-3SFT) synthesized by using 1 mol% Ni(dppp)Cl_2_ catalyst, has Mn = 25,600, Mw = 36,200, which are roughly 2.5 times the Mn and Mw of P(3HT-*b*-3SFT) synthesized by using 2 mol% Ni(dppp)Cl_2_ catalyst. This result suggests that the molecular weight of copolymers could be controlled by the amount of Ni(dppp)Cl_2_.

### 2.3. Film Characterization of Polymer

Thin films of P(3HT-*b*-3SFT) block copolymers and the P3HT homopolymer were fabricated to investigate their optical properties and surface morphologies. Thin films of polymers were prepared by spin coating from *o*-dichlorobenzene (ODCB) on quarts substrates. In the UV-Vis spectra, P(3HT-*b*-3SFT)s, prepared by the 1 mol% and 2 mol% Ni(dppp)Cl_2_ catalysts, and P3HT show the maximum absorption (λ_max_) at 526, 524 and 556 nm, respectively, with a shoulder peak at approximately 600 nm as indicated in Figure 3. The P3SFT homopolymer film has been reported to show λ_max_ of 482 nm [22]. Even though the content of P3SFT in P(3HT-*b*-3SFT) is small, the influence of P3SFT on optical property of P(3HT-*b*-3SFT) is so significant, that the λ_max_ value of P(3HT-*b*-3SFT) shifts toward the λ_max_ of P3SFT homopolymer.

The surface morphology of the thin film of P3HT and P(3HT-*b*-3SFT)s were observed by the atomic force microscopy (AFM). Figure 4 shows AFM phase images of thin films of P3HT and P(3HT-*b*-3SFT). Roughness values for all polymers obtained from AFM images are summarized in Table 2. Similar roughness values for P3HT and P(3HT-*b*-3SFT)s were obtained, whereas the phase image of P(3HT-*b*-3SFT) was found to be quite different from that of P3HT. The phase image of the P3HT film shows a homogeneous surface, while the P(3HT-*b*-3SFT) film shows round-shape domains on the surface. These domains are apparently obtained due to the phase separation of the hydrocarbon and fluorinated carbon segments by the repulsive nature of the fluorine atom (Figure 5); and the difference of the domain size is caused by the molecular weight of the copolymer as well as the content of P3SFT in P(3HT-*b*-3SFT). These results suggest that even the small P3SFT segment of P(3HT-*b*-3SFT) is enough to influence the morphology of the polymer thin film.

### 2.4. Properties of Photovoltaic Cells

The BHJ solar cells based on the blends of P(3HT-*b*-3SFT) and [6,6]-phenyl-C_61_-butyric acid methyl ester (PCBM) were fabricated and the solar cell properties were characterized. The device structure was glass/ITO/PEDOT:PSS/blend of P(3HT-*b*-3SFT) and PCBM/Al. The property of solar cells was measured by using a solar simulator (100 mW/cm^2^, AM 1.5). We fabricated the solar cells with P(3HT-*b*-3SFT) (1 mol% and 2 mol% Ni(dppp)Cl_2_):PCBM (1:1 by weight) which were annealed at 100 °C for 20 min. Figure 6 shows the current density-voltage characteristics of the BHJ solar cells. The corresponding photovoltaic parameters (short circuit current density *J*_sc_, open circuit voltage *V*_oc_, fill factor *FF* and solar cell efficiency *E_ff_*) are summarized in Table 3. The device with P(3HT-*b*-3SFT) (1 mol% Ni(dppp)Cl_2_) exhibits higher *J*_sc_ and *FF* values than that with P(3HT-*b*-3SFT) (2 mol% Ni(dppp)Cl_2_). On the other hand, the *V*_oc_ value of the solar cell with P(3HT-*b*-3SFT) (2 mol% Ni(dppp)Cl_2_) was higher than that with P(3HT-*b*-3SFT) (1 mol% Ni(dppp)Cl_2_). The surface morphology of the solar cells by AFM was then studied. The phase image of P(3HT-*b*-3SFT) (1 mol% Ni(dppp)Cl_2_) has smaller domains (average domain area:0.006 μm) than the P(3HT-*b*-3SFT) (2 mol% Ni(dppp)Cl_2_) (average domain area:0.012 μm). This result is contrary to the AFM phase image of only P(3HT-*b*-3SFT) shown in Figure 5, and the solar cell which has smaller domain shows better solar cell performance. It seems that the blend of PCBM interrupts aggregation of diblock copolymers, as a result the domain size of copolymers for solar cells is smaller than those of copolymer thin films. However we cannot ascertain why the domain size of P(3HT-*b*-3SFT) (1 mol% Ni(dppp)Cl_2_) is smaller than that of P(3HT-*b*-3SFT) (2 mol% Ni(dppp)Cl_2_).

We also fabricated the solar cells with P(3HT-*b*-3SFT) (1 mol% Ni(dppp)Cl_2_), annealed at 140 °C, and data were compared with the non-annealed version. The current density-voltage characteristics of these BHJ solar cells are shown in Figure 7. The corresponding photovoltaic parameters are summarized in Table 4. In our previous study [26], the best annealing temperature for P3HT/PCBM solar cells was 100 °C. However, the non-annealed solar cell with P(3HT-*b*-3SFT) showed best performance with *J*_sc_ = 4.10 mA/cm^2^, *V*_oc_ = 0.58 V, *FF* = 0.35, *E_ff_* = 0.84%.

Figure 8 shows the AFM images of morphology for solar cells with P(3HT-*b*-3SFT)/PCBM prepared under various annealing conditions. The AFM images of the solar cells annealed at 100 °C and 140 °C showed round shape domains, and domains of the device annealed at 140 °C are larger than at 100 °C. Since these domains disturb formation of the bicontinuous network in the BHJ solar cells, the self assembly of P(3HT-*b*-3SFT) decrease solar cells properties by annealing.

## 3. Experimental Section

### 3.1. Material and Instrumentation

Isopropylmagnesium Chloride in Tetrahydrofuran, (1 mol/L) were purchased from Tokyo Chemical Industry Co., Ltd. Ni(dppp)Cl_2_ was purchased from Sigma-Aldrich Co. 2,5-dibromo-3-hexylthiophene and 2,5-dibromo-3-(4,4,5,5,6,6,7,7,7-nonafluoroheptyl)thiophene were synthesized by previously reported methods [22,25].

^1^H and ^19^F NMR spectra in CHCl_3_ were measured using a Varian Gemini-200, 300 and ^1^H and ^13^C NMR spectra in CHCl_3_ for polymers were measured using Bruker AV-500. Molecular weight (Mn, Mw, Mw/Mn) were determined by Tosoh Gel Permeation Chromatography (GPC) with a UV detector using THF as the eluent at 40 °C. UV-Vis spectra of thin films were recorded using a JASCO V-570. Atomic Force Microscopy (AFM) images were done with a JEOL JSM-5600 scanning electron microscope operating in tapping mode. The current-voltage (*J*-*V*) measurements of the polymer photovoltaic cell were carried out using a solar simulator under the illumination of AM 1.5, 100 mW/cm^2^.

### 3.2. Synthesis of Poly(3-hexylthiophene)-*b*-poly(3-(4,4,5,5,6,6,7,7,7-nonafluoroheptyl)thiophene) *(10)*

All glass apparatuses were dried prior to use. Two round bottomed flasks equipped with a three-way stopcock were dried by heating under reduced pressure and cooled to room temperature under Ar. 2,5-dibromo-3-hexylthiophene (D3HT) (6) (400 mg, 1.23 mmol) was placed in one of the flasks, and 2,5-dibromo-3-(4,4,5,5,6,6,7,7,7-nonafluoroheptyl)thiophene (D3SFT) (308 mg, 0.62 mmol) (5) was placed in the other. They were then evacuated under reduced pressure to remove any water and oxygen inside. Dry THF (7.0 mL) was added into the D3HT flask (1), and the solution was stirred at 0 °C. Isopropyl magnesium chloride (1.0 M solution in THF, 1.23 mL, 1.23 mmol) was added to the solution, and the mixture was heated to reflux under Ar (7). After 45 min, a suspension of Ni(dppp)Cl_2_ (13.3 mg, 0.025 mmol, 2.0 mol%) in dry THF (8.0 mL) was added, and the reaction mixture was heated to reflux for 1 h.

Dry THF (3.0 mL) was added to the other flask for D3SFT (5), and the solution was stirred at 0 °C. Isopropylmagnesium chloride (1.0 M solution in THF, 0.62 mL, 0.62 mmol) was added to the solution, and the mixture was stirred at reflux under argon for 45 min. This mixture (9) was added to the polymerization mixture of D3HT (8) via a syringe. The mixture was stirred at reflux under Ar for 1 h. The reaction mixture was cooled to room temperature, and then poured into methanol (100 mL) and residue was filtered and purified via Soxhlet extraction successively with methanol, acetone, and chloroform. The chloroform fraction was concentrated under vacuum to give P(3HT-*b*-3SFT) as a purple solid (138.6 mg, 33.3%) (10). P(3HT-*b*-3SFT) synthesized by using 1.0 mol% Ni(dppp)Cl_2_, afforded a 30.0% yield.

### 3.3. Film Preparation for Measurement of UV-Spectrum and AFM

To investigate morphology and the optical properties of P(3HT-*b*-3SFT)s and P3HT as a reference, thin films of the polymers were prepared by spin coating from *o*-dichlorobenzene on quarts substrates at room temperature, then annealed at 140 °C for 10 min inside a N_2_-filled glove box. Measurement of AFM and UV-Vis spectroscopy was carried out on the same sample.

### 3.4. Fabrication and Measurement of Solar Cells

The indium tin oxide (ITO)-coated glass substrate was cleaned successively with acetone and methanol under ultrasonication for 5 min, and cleaned by nitrogen gas. Then the substrate was cleaned by ultraviolet ozone treatment for 1 h. Poly(3,4-ethylenedioxythiophene):poly(styrenesulfonate) (PEDOT:PSS) (Baytron P AL 4083, HC Starck) was spin-coated on ITO at 2,000 rpm in air. Then the device was transferred to the N_2_-filled glove box, and dried at 100 °C for 5 min. The polymer/PCBM mixture was prepared by dissolving together in ODCB (30 mg/mL, 1:1 wt:wt) and stirring overnight. The active layer of the device was formed by spin casting at 2,000 rpm from the mixture on the PEDOT/PSS layer. Then the films were annealed at 100 °C or 140 °C, each for 20 min. The top electrode of Al was deposited on the active layer by a vacuum deposition. Then the device was annealed at 140 °C for 10 min inside a N_2_-filled glove box.

## 4. Conclusions

We have synthesized poly[(3-hexylthiophene)-*block*-(3-(4,4,5,5,6,6,7,7,7-nonafluoroheptyl) thiophene)] (P(3HT-*b*-3SFT)) by the GRIM, coupled with nickel-catalyzed coupling polymerization of D3HT followed by D3SFT, which were composed of P3HT and marginal P3SFT. Even though the amount of P3SFT is very small, it had a significant influence on the property of P(3HT-*b*-3SFT).

We also fabricated solar cells based on the blends of P(3HT-*b*-3SFT)s and PCBM, which showed phase separation as expected. The solar cells based on P(3HT-*b*-3SFT)s, synthesized by using 1 mol% Ni(dppp)Cl_2_, indicated better photovoltaic properties than those based on P(3HT-*b*-3SFT)s (2 mol% Ni(dppp)Cl_2_). This result may be due to the difference of domain size in the active layer, and the solar cell based on P(3HT-*b*-3SFT) (1 mol% Ni(dppp)Cl_2_) is smaller. In addition, we investigated the influence of annealing temperatures on the performance of solar cells and found that the annealing process induced formation of large domains, and the properties of the annealed device were decreased.

Based on this study, we will study the solar cell composed of P(3HT-*b*-3SFT) and fullerene derivatives with perfluoroalkyl substituents, which is expected to have a different morphology due to the interactive effects of both perfluoro chains.

## Figures and Tables

**Figure 1.** The image of self-assembly of diblock copolymer with semifluorinated carbon and hydrocarbon segments and PCBM on crystallization.

**Figure 2.** GPC charts of P(3HT-*b*-3SFT) synthesized by using Ni(dppp)Cl_2_ (1 mol% and 2 mol%).

**Figure 3.** UV-Vis spectra of thin films of P(3HT-*b*-3SFT)s synthesized by using Ni(dppp)Cl_2_ (1 mol% and 2 mol%) and P3HT.

**Figure 4.** AFM phase images. (**a**) P3HT film; (**b**) P(3HT-*b*-3SFT) film (image size: 1 μm × 1 μm).

**Figure 5.** The model image of phase separation of P(3HT-*b*-3SFT).

**Figure 6.** *J*-*V* characteristics of polymer solar cells with PCBM:P(3HT-*b*-3SFT)s.

**Figure 7.** *J*–*V* characteristics and spectral responsivity of polymer solar cells with PCBM:P(3HT-*b*-3SFT) synthesized by using 1 mol% Ni(dppp)Cl_2_.

**Figure 8.** AFM phase images of the solar cells with PCBM:P(3HT-*b*-3SFT). (**a**) non-annealed; (**b**) 100 °C; (**c**) 140 °C (image size: 1 μm × 1 μm).

**Scheme 1.** Synthetic route for 2,5-dibromo-3-(4,4,5,5,6,6,7,7,7-nonafluoroheptyl)thiophene.

**Scheme 2.** Synthetic route for poly[(3-hexylthiophene)-*block*-(3-(4,4,5,5,6,6,7,7,7-nonafluoroheptyl)thiophene)].

**Table 1.** Summary of GPC measurements of P3HT prepolymer and diblock copolymer, P(3HT-*b*-3SFT).

**Polymer**	**Mn**	**Mw**	**Mw/Mn**
P(3HT-*b*-3SFT) (1 mol% Ni(dppp)Cl_2_)	25,600	36,200	1.4
P(3HT-*b*-3SFT) (2 mol% Ni(dppp)Cl_2_)	10,500	13,500	1.2

**Table 2.** The roughness of films from atomic force microscopy (AFM) analysis.

**Polymer**	**Ra (nm)**	**RMS (nm)**	**Average Domain Area in Phase Image (μm^2^)**
P3HT	1.22	1.51	-
P(3HT-*b*-3SFT) (1 mol% Ni(dppp)Cl_2_)	2.03	2.80	0.050
P(3HT-*b*-3SFT) (2 mol% Ni(dppp)Cl_2_)	1.98	2.58	0.019

**Table 3.** The characteristics of polymer solar cells with P(3HT-*b*-3SFT).

**Materials**	***V***_**oc**_**(V)**	***J***_**sc**_**(mA/cm^2^)**	***FF***	***E****_ff_***(%)**
PCBM:P(3HT-*b*-3SFT) (1 mol% Ni(dppp)Cl_2_)	0.54	3.42	0.28	0.52
PCBM:P(3HT-*b*-3SFT) (2 mol% Ni(dppp)Cl_2_)	0.59	2.65	0.23	0.35

**Table 4.** The characteristics of polymer solar cells with P(3HT-*b*-3SFT).

**Annealing Temp**	***V***_**oc**_**(V)**	***J***_**sc**_**(mA/cm^2^)**	***FF***	***E****_ff_***(%)**
R.T.	0.58	4.10	0.35	0.84
100 °C	0.54	3.42	0.28	0.52
140 °C	0.41	2.27	0.23	0.21
